The article "PET/CT Evaluation of the Effect of Allogeneic Hematopoietic Stem Cell Transplantation in the Treatment of T-Cell Lymphoblastic Lymphoma" was published in 2022. Journal: Contrast Media Mol Imaging.

# PET/CT Evaluation of the Effect of Allogeneic Hematopoietic Stem Cell Transplantation in the Treatment of T-Cell Lymphoblastic Lymphoma

**DOI:** 10.1155/2022/6057017

**Published:** 2022-08-16

**Authors:** Jin Zhao, Xiaojing Guo, Li Ma, Meijing Zheng, Tao Guan, Liping Su

**Affiliations:** Department of Hematology, Shanxi Province Cancer Hospital, Shanxi Hospital Affiliated to Cancer Hospital, Chinese Academy of Medical Sciences, Cancer Hospital Affiliated to Shanxi Medical University, Taiyuan 030013, Shanxi, China

## Abstract

The aim of this study was to investigate the clinical value of positron emission tomography/computerized tomography scanning (PET/CT) in the evaluation of the effect of allogeneic hematopoietic stem cell transplantation in the treatment of T lymphoblastic lymphoma. 12 relevant research articles were collected through layer-by-layer screening in large databases such as Pubmed, Baidu Scholar, and China How Net, and analyzed and summarized using indicators such as progression-free survival (PFS), overall survival (OS), hazard ratio (HR), maximum standardized uptake value (SUV max), total metabolic tumor volume (TMTV), total lesion glycolysis (TLG), elevated lactate dehydrogenase (LDH), and *β*2-microglobulin (*β*2-MG). The results showed that before treatment, ^18^F-FDG PET/CT baseline diagnosis could accurately stage the patients; during treatment, ^18^F-FDG PET/CT detection could provide effective treatment information; and after treatment, complications were found during ^18^F-FDG PET/CT detection. In summary, ^18^F-FDG PET/CT can monitor and evaluate treatment prognosis at baseline, middle, and late stages, and ^18^F-FDG PET/CT has become an indispensable and important examination technique in clinical work.

## 1. Introduction

According to different lymphoblastic lymphomas of cellular origin, they can be divided into two groups: T-cell lymphoblastic lymphoma and B-cell lymphoblastic lymphoma (B-LBL), as shown in Figure 1 [1, 2]. The probability of occurrence of T-cell lymphoblastic lymphoma disorders accounts for about 90% of all lymphoblastic lymphoma disorders and is currently the focus of clinical research [3]. At present, T-cell lymphoblastic lymphoma and T-cell acute lymphocytic leukemia (T-ALL) are defined as the same type of disease in clinical practice [4, 5]. T-cell lymphoblastic lymphoma is a rare and highly aggressive Hodgkin's lymphoma in clinical practice, which is common in children and adolescents, especially in male children and adolescents [6, 7]. At present, the treatment for T-cell lymphoblastic lymphoma in clinical practice is mainly high-dose chemotherapy (HDC) combined with a variety of drugs [8–10]. However, clinical studies have shown that although the progression-free survival (PFS) of patients treated with chemotherapy reaches more than 50%, there is still a probability of recurrence of about 35% [11]. With the continuous clinical exploration of research experts, it has been found that allogeneic hematopoietic stem cell transplantation can play a better role in patients with aggressive lymphoma who fail to respond to chemotherapy and are resistant [12, 13]. It can not only improve the survival probability of patients but also reduce the probability of recurrence in the early stage of treatment, especially for patients in the early stage of the disease [14, 15]. However, some experts have proposed that patients with T-cell lymphoblastic lymphoma still have a high cumulative recurrence rate (CIR) after hematopoietic stem cell transplantation [16, 17]. In order to better explore the clinical and therapeutic effects of allogeneic hematopoietic stem cell transplantation, a number of studies have used positron emission tomography/computerized tomographic scanning (PET/CT) for efficacy evaluation [18]. Studies have shown that ^18^F-FDG PET/CT before and after allogeneic hematopoietic stem cell transplantation is a predictor of overall survival (OS) and disease-free survival (DFS) in acute leukemia (AL) [19, 20].

The article "PET/CT Evaluation of the Effect of Allogeneic Hematopoietic Stem Cell Transplantation in the Treatment of T-Cell Lymphoblastic Lymphoma" was published in 2022. Journal: Contrast Media Mol Imaging.

In summary, the literature on the prognostic evaluation of allogeneic hematopoietic stem cell transplantation for T-cell lymphoblastic lymphoma by baseline examination, interim examination, and ^18^F-FDG PET/CT scan after treatment was collected, analyzed, and summarized. It was to further understand the application value of PET/CT in the evaluation of the effect of allogeneic hematopoietic stem cell transplantation in the treatment of T lymphoblastic lymphoma, providing more reference for hematopoietic stem cell transplantation in the treatment of T lymphoblastic lymphoma.

## 2. Materials and Methods

This study aimed to explore the prognostic effect of 18F-FDG PET/CT scanning in T lymphoblastic lymphoma at baseline, mid-term, and posttreatment of allogeneic hematopoietic stem cell transplantation. The articles on the applicability of 18F-FDG PET/CT scans, allogeneic hematopoietic stem cell transplantation, and T lymphoblastic lymphoma patients were reviewed. The research and selection process of related articles are shown in Figure 2. It searched large databases such as Pubmed, Baidu Scholar, China HowNet, etc., to improve the probability of getting the best search results. According to previous research experience [21, 22], it needed to query documents in multiple databases. Because there was no database that could record all the literature, it needed to supplement the related literature in another database [23].

The article "PET/CT Evaluation of the Effect of Allogeneic Hematopoietic Stem Cell Transplantation in the Treatment of T-Cell Lymphoblastic Lymphoma" was published in 2022. Journal: Contrast Media Mol Imaging.

Inclusion criteria were defined as follows: (1) literature written in English and published in conferences or journals; and (2) the main research topic of the literature was the prognostic value of 18F-FDG PET/CT before and after allogeneic hematopoietic stem cell transplantation for T lymphoblastic lymphoma.

The above research was mainly a case-control analysis, including the diagnosis, detection, and follow-up of patients with T lymphoblastic lymphoma after treatment. Through the identification and selection of articles in Figure 2, a total of 100 articles were collected from various scientific searches in the process of research and paper query. Afterwards, the articles were classified as available or unavailable by browsing the contents of the abstract and conclusion sections, among which 70 articles with irrelevant and duplicate records were excluded. After that, the remaining 30 articles were read throughout, and 18 articles were excluded. Finally, a total of 12 research papers met the requirements and were used for this research analysis.

The value of ^18^F-FDG PET/CT scanning in the detection of T-lymphocytic lymphoma at baseline, mid-term, and posttreatment of allogeneic hematopoietic stem cell transplantation was analyzed by collecting PFS, OS, hazard ratio (HR), maximum standardized uptake value (SUV max), total metabolic tumor volume (TMTV), total lesion glycolysis (TLG), elevated lactate dehydrogenase (LDH), and *β*2-microglobulin (*β*2-MG).

## 3. Literature Overview

### 3.1. Role of Baseline ^18^F-FDG PET/CT Assessment

After long-term clinical practice, it has been confirmed that the treatment of various diseases is often closely related to the accuracy of diagnosis, especially tumor diseases. Different benign and malignant tumors and stages of tumor disease can have an impact on treatment options. Therefore, baseline ^18^F-FDG PET/CT scanning for patients with T-cell lymphoblastic lymphoma before treatment has been widely used in clinical practice. The extent of lesion involvement in patients with T-cell lymphoblastic lymphoma is determined by ^18^F-FDG PET/CT detection for definitive staging to develop an accurate treatment plan while evaluating the prognosis of patients. Zou et al. [24] pointed out that ^18^F-FDG PET/CT has quite high accuracy in the identification of malignant lymphoma and high clinical application value. Feng et al. [25] investigated the optimal prognostic model for T-cell lymphoblastic lymphoma in 37 initial treatment patients with T-cell lymphoblastic lymphoma who underwent PET-CT scanning. The results showed that the optimal cut-off values of SUV max, TMTV, and TLG were 12.7, 30^2^ cm^3^, and 890, respectively, and high SUV max, TMTV, and TLG indicated that PFS and OS were shortened. It can be observed that baseline ^18^F-FDG PET/CT detection can be used to predict the prognosis of T-cell lymphoblastic lymphoma disease, of which the main predictors are SUV max, TMTV, and TLG, and baseline SUV max, TMTV, and TLG can provide a strong prediction for patients with poor prognosis. Alternatively, Becker et al. [26] carried out an experiment about the predictive value of baseline ^18^F-FDG PET/CT in patients with T-cell lymphoblastic lymphoma, and 36 patients with T-cell lymphoblastic lymphoma were studied. The results showed that the cut-off value of SUV max (8.76) could predict 3-year PFS, and the cut-off value of 80% ΔSUV max could predict 3-year OS, further suggesting that ^18^F-FDG PET/CT detection is helpful to predict the therapeutic effect of patients, of which the main outcome measure is SUV max. The lower initial SUV max indicates that the treatment prognosis of patients with T-cell lymphoblastic lymphoma will be poor. Li et al. [27] further explored the value of ^18^F-FDG PET/CT, and the results showed that pretreatment SUV max ≥9.5, disease stages II and III-IV, LDH, and *β*2-MG were most strongly associated with unfavorable PFS and OS. Based on the above studies, baseline 18F-FDG PET/CT can not only accurately diagnose the staging of T lymphoblastic lymphoma patients, but also effectively predict the prognosis of patients. The results of the baseline 18F-FDG PET/CT prediction study are shown in Table 1. Table 1 showed that the baseline SUV max value had certain application advantages.

The article "PET/CT Evaluation of the Effect of Allogeneic Hematopoietic Stem Cell Transplantation in the Treatment of T-Cell Lymphoblastic Lymphoma" was published in 2022. Journal: Contrast Media Mol Imaging.

### 3.2. Role of Interim ^18^F-FDG PET/CT Evaluation

In recent years, many experts have paid attention to the study of interim ^18^F-FDG PET/CT detection and evaluation in the prognosis of lymphoma treatment. The use of interim ^18^F-FDG PET/CT in the examination of patients during treatment can not only obtain the response of the lesion to the treatment method to adjust the treatment plan as early as possible, but also evaluate the prognosis of patients. As a highly concerning allogeneic hematopoietic stem cell transplantation treatment in clinical practice, its therapeutic effect in T-cell lymphoblastic lymphoma is also the focus of clinical attention. The sensitivity and adverse reactions of allogeneic hematopoietic stem cell transplantation in the treatment of patients with T-cell lymphoblastic lymphoma require clinical exploration. Relevant studies have shown that allogeneic hematopoietic stem cell transplantation is a safe and effective method for the treatment of T-cell lymphoblastic lymphoma, with a recurrence rate of 20% after transplantation, which is significantly lower than the previous 50%, with a complete remission (CR) rate of 63%, and a 3-year OS of 56.2% [28]. However, there are still risk events during allogeneic hematopoietic stem cell transplantation that attract the attention of clinical experts. After all, it poses a certain threat to the safety of patients. For example, Longhitano et al. [29] put forward that for immunocompromised patients, there was a risk of fungal and bacterial infections during allogeneic hematopoietic stem cell transplantation with a high mortality rate. It was proposed that FDG PET/CT detection can be used for the diagnosis and monitoring of complex infections in immunocompromised patients, which played a key role in guiding the decision of treatment duration and suggested the necessity of surgical intervention. Williams et al. [30] performed the exploration in 23 patients with hematological malignancies who underwent HSCT and evaluated the effect of ^18^F-fluorothymidine (^18^F-FLT) PET/CT. The results showed that ^18^F-FLT allows the quantification and tracking of human subclinical bone marrow repopulation and can reflect the biological basis for hematopoietic stem cell (HSC) recovery after HSCT. It was proposed that the uptake of ^18^F-FDG in tumor tissue was higher than that of ^18^F-FLT [31]. Therefore, ^18^F-FDG PET/CT reflects the therapeutic effect of patients. Thus, ^18^F-FDG PET/CT is able to detect various body responses to this treatment during allogeneic hematopoietic stem cell transplantation treatment and facilitate further clinical treatment. Dai et al. [32] used the improved ^18^F-FDG PET/CT technique to evaluate the prognosis after stem cell transplantation, and found that the improved ^18^F-FDG PET/CT technique had a high application value in predicting PFS and OS in patients after stem cell transplantation treatment, especially in patients after 3 to 6 months of treatment. However, some experts proposed that for patients with relapsed or refractory T-lymphocytic lymphoma, ^18^F-FDG PET/CT is used to predict the treatment prognosis after HSCT [33]. ^18^F-FDG PET/CT cannot well predict the OS of patients, but there is a strong correlation between the detection results and PFS, indicating that ^18^F-FDG PET/CT detection can effectively guide the subsequent clinical treatment options. Ying et al. [34] presented that, based on multivariate analysis, HSC transplantation after HDC treatment could predict survival using ^18^F-FDG PET/CT detection in patients with lymphoma. Based on the above content, ^18^F-FDG PET/CT can not only effectively monitor various reactions (drug sensitivity, adverse reactions, etc.) of patients during HSC transplantation but also predict the prognosis of patients after receiving HSC transplantation, which has good clinical value.

The article "PET/CT Evaluation of the Effect of Allogeneic Hematopoietic Stem Cell Transplantation in the Treatment of T-Cell Lymphoblastic Lymphoma" was published in 2022. Journal: Contrast Media Mol Imaging.

The results of the application study of ^18^F-FDG PET/CT prediction in the mid-treatment period were shown in Table 2.

### 3.3. Role of Late ^18^F-FDG PET/CT Evaluation

Staged diagnosis and evaluation of prognosis of T-cell lymphoblastic lymphoma before treatment, evaluation of the treatment process, and evaluation of treatment response have a significant impact on the treatment of patients and have certain importance. However, it is also very important to reexamine the patients after treatment to monitor their survival status. Although most patients with T-cell lymphoblastic lymphoma receiving allogeneic hematopoietic stem cell transplantation can be cured, some adult patients with lymphoblastic lymphoma will develop drug resistance after first-line treatment and even have a recurrence. Therefore, clinical studies mainly observe the PFS, OS, complications, and recurrence of the disease in patients after treatment. Some researchers have proposed that recurrence of acute lymphocytic leukemia (ALL) remains the leading cause of death from hematologic malignancies after allogeneic hematopoietic stem cell transplantation, especially for patients with high-risk cytogenetic or molecular abnormalities [35]. Therefore, reexamination after treatment is very necessary for the monitoring of the patient's condition. Isik et al. [36] used PET scans at baseline, interim, and posttreatment to predict prognosis in pediatric Hodgkin's lymphoma and concluded that SUV max by PET scans is effective in predicting 3-year PFS in patients at the end of treatment. These results indicate that ^18^F-FDG PET/CT can be used to predict the survival of patients with Hodgkin's lymphoma after HSC transplantation therapy. As a serious complication after solid organ and HSC transplantation, posttransplantation lymphoproliferative disease is also the focus of detection after treatment. Posttransplantation lymphoproliferative disease is closely related to the morbidity and mortality of patient treatment. Montes et al. [37] analyzed the value of CT, magnetic resonance imaging (MRI), and ^18^F-FDG PET/CT in the diagnosis of patients with posttransplantation lymphoproliferative disease or in the assessment of treatment response. It revealed that FDG-PET/CT found 27.8% of posttransplant lymphoproliferative lesions undetected by CT and/or MRI techniques, and FDG-PET/CT is one of the most frequently used imaging modalities by clinical researchers in the diagnostic study of patients with posttransplantation lymphoproliferative disease at this stage. Kim and Kim [38] analyzed the diagnostic performance of ^18^F-FDG PET/CT or PET/CT for the detection of posttransplantation lymphoproliferative disease. It showed that the overall diagnostic odds ratio of ^18^F-FDG PET/CT or PET/CT was 83 and the area under the curve was 0.96, suggesting that ^18^F-FDG PET/CT or PET/CT has high sensitivity and specificity for the diagnosis of posttransplant lymphoproliferative lesions, but the accuracy needs further confirmation. Regarding relapse of ALL, Hunger and Raetz [39] mentioned that the treatment of relapsed ALL in children is clinically challenging and that the survival rate of children after relapse will be greatly reduced compared with that observed in initial diagnosis, which is related to the failure to be detected in a timely manner. Therefore, it is necessary to detect relapse in patients with T-cell lymphoblastic lymphoma after treatment, especially in critically ill patients. Berriolo-Riedinger et al. [40] pointed out that PET-CT has become the gold standard imaging technique at the end of treatment for Hodgkin's lymphoma at this stage. When PET-CT results are negative, it indicates that the patient's tumor lesions have reached the degree of complete remission. However, there is a lack of clinical studies on the evaluation of ^18^F-FDG PET/CT for recurrence in patients with T-cell lymphoblastic lymphoma after allogeneic hematopoietic stem cell transplantation. Therefore, ^18^F-FDG PET/CT in this area needs further exploration. Through the above studies, ^18^F-FDG PET/CT has a considerable effect in reexamination and monitoring of patients with T-cell lymphoblastic lymphoma after treatment, but the detection value for the situation after recurrence requires clinical in-depth exploration. The results of the application study of ^18^F-FDG PET/CT prediction after treatment were shown in Table 3.

The article "PET/CT Evaluation of the Effect of Allogeneic Hematopoietic Stem Cell Transplantation in the Treatment of T-Cell Lymphoblastic Lymphoma" was published in 2022. Journal: Contrast Media Mol Imaging.

## 4. Application Basis and Background of ^18^F-FDG PET/CT

With the rapid development of PET technology in recent years, the use of various radioactive molecular tracers to display the molecular metabolism, receptors, and nerve distribution of the body has become the most advanced molecular imaging technology. PET examination technology can display the physiological metabolism of human tissues, organs, and lesions, but its image clarity is poor, which is not conducive to clinical disease assessment. In the early 1990s, the technology of combining radiomics in the field of radiology was relatively mature, and it was widely combined with CT technology. CT scanning can not only locate the lesions, but also has better image quality than PET, thus making up for the shortcomings of PET imaging. Therefore, PET/CT is an examination technology that combines the function display effect of PET with the anatomical structure display effect of CT. PET/CT is equivalent to combining the advantages of both. Studies have shown that PET/CT has high sensitivity and specificity in disease detection, and the images are clearly displayed, which is convenient for doctors to diagnose, stage, and evaluate the efficacy of the disease [41, 42]. Studies have shown that PET plays a crucial role in the accurate staging and recurrence assessment of lymphoma, and the improved fluorodeoxyglucose (FDG)-PET/CT fusion has improved the prognosis of lymphoma patients [43]. ^18^F-FDG plays an important role in the PET/CT scanning process. As one of the most common tracers in PET/CT scans, ^18^F-FDG can reflect the severity and prognosis of a patient's tumor disease through the uptake intensity. Among them, the semi-quantitative parameter in 18F-FDG images, the maximal standardized uptake value (SUVmax), is one of the main indicators to evaluate the tumor condition. The preparation and application process of ^18^F-FDG drug was shown in Figure 3. The imaging principle of 18F-FDG PET/CT is shown in Figure 4.

Dai et al. [44] proposed that the sensitivity, specificity, positive predictive value, negative predictive value, and accuracy of ^18^F-FDG PET-CT in patients undergoing allogeneic hematopoietic stem cell transplantation were 100%, 92.2%, 75.0%, 100%, and 93.7%, respectively. Moreover, it can be used to evaluate the progression-free survival (PFS) of patients, which can provide an important basis for the selection of subsequent treatment options for patients with lymphoblastic lymphoma. El-Galaly et al. [45] also proposed that FDG-PET/CT plays an important role in all stages of lymphoma and is a key step to improving and enhancing the targeted treatment of lymphoma. Therefore, 18F-FDG PET/CT has good accuracy and clinical application value in evaluating the effect of allogeneic hematopoietic stem cell transplantation in T lymphoblastic lymphoma.

## 5. Challenges and Limitations

Through recent studies, it has been found that 18F-FDG PET/CT imaging technology has a good application effect in evaluating the effect of allogeneic hematopoietic stem cell transplantation in the treatment of T lymphoblastic lymphoma. However, its application effect is different at different treatment intervals, and the main effect is also different. In order to make PET/CT imaging technology reach a higher level in clinical diagnosis and evaluation of treatment effects and continuous exploration is required. The specific limitations are shown in Table 4. According to the content in the table, the specific application deficiencies include the following aspects:

- There is a significant difference in the evaluation results of the disease when the tracer is used alone and in combination;
- ^18^F-FDG PET/CT evaluation has a limited treatment window;
- the prognosis after HSCT application cannot be predicted before treatment;
- there are false positive results;
- the literature on postassessment studies is lacking and needs to be expanded.

The article "PET/CT Evaluation of the Effect of Allogeneic Hematopoietic Stem Cell Transplantation in the Treatment of T-Cell Lymphoblastic Lymphoma" was published in 2022. Journal: Contrast Media Mol Imaging.

It should further explore and improve the application of ^18^F-FDG PET/CT based on the shortcomings of the above studies, so as to provide patients with more effective inspection methods.

## 6. Conclusions

By summarizing the above contents, baseline, interim, and late ^18^F-FDG PET/CT detection has a good effect in evaluating the prognosis of T-cell lymphoblastic lymphoma treated with allogeneic hematopoietic stem cell transplantation, and it has been verified and recognized by many experts. Baseline ^18^F-FDG PET/CT diagnosis for patients with T-cell lymphoblastic lymphoma before treatment can accurately stage the patients and improve the diagnostic level. During treatment, the use of interim ^18^F-FDG PET/CT detection for real-time detection of treatment response in patients with T-cell lymphoblastic lymphoma can provide effective treatment information and facilitate doctors to improve the treatment plan; after treatment, the use of late ^18^F-FDG PET/CT detection for patients can timely detect complications and facilitate timely treatment.

Combined with the above content, baseline, mid-term, and late ^18^F-FDG PET/CT can monitor and evaluate the prognosis of treatment, and ^18^F-FDG PET/CT has become an indispensable and important examination technique in clinical work. However, how to improve the monitoring accuracy of ^18^F-FDG PET/CT in disease recurrence still needs further exploration.

## Figures and Tables

**Figure 1:** Classification of lymphoblastic lymphoma.

**Figure 2:** The flow chart of a literature search.

**Figure 3:** Preparation and application process of the ^18^F-FDG drug.

**Figure 4:** The imaging principle of ^18^F-FDG PET/CT.

**Table 1:** Baseline 18F-FDG PET/CT prediction study results statistics.

References	Research results	Conclusion
Reference [25]	The optimal cut-off values of SUV max, TMTV, and TLG were 12.7, 302 cm^3^, and 890, respectively; and both PFS and OS were shortened with increasing.	SUVmax, TMTV, and TLG predict T-LBL worsening

Reference [26]	SUVmax ≤8.76 predicted 3-year event-free survival of 31.6% and overall survival of 35.0%	Low initial SUV max predicts poorer prognosis.

Reference [27]	SUVmax ≥9.5, disease stage II and III-IV, elevated LDH, elevated *β*2-MG	Strongest correlation with PFS and OS

The article "PET/CT Evaluation of the Effect of Allogeneic Hematopoietic Stem Cell Transplantation in the Treatment of T-Cell Lymphoblastic Lymphoma" was published in 2022. Journal: Contrast Media Mol Imaging.

**Table 2:** Statistics of interim ^18^F-FDG PET/CT prediction study results.

References	Research results	Research conclusion
Reference [29]	^18^F-FDG PET/CT facilitated complete recovery and transition to HCT in two patients.	FDG-PET/CT had a new role in the diagnostic and surveillance pathways of complex infections in high-risk immunocompromised patients.

Reference [30]	There was a significant difference in ^18^F-FLT intensity between pre-HSCT myeloablative infusion and subclinical stellate recovery (*p* = 0.00031).	^18^F-FLT allowed quantification and tracking of human subclinical bone marrow regeneration and reveals new insights into the biology of stellate cell recovery after HSCT.

Reference [31]	The sensitivity of FLT-PET/CT was lower than that of FDG-PET/CT	The uptake of 18F-FDG in tumor tissue was higher than that of ^18^F-FLT

Reference [32]	ASCT ^18^F-FDG positivity after PET-CT was associated with lower PFS and OS; PET-CT outcome was the only independent factor associated with OS (*p* = 0.028); PET within 3–6 months after ASCT-In patients with CT scan, the PFS and OS prognosis were better in the PET-CT negative group	^18^F-FDG PET/CT technology had high application value in predicting PFS and OS of patients after stem cell transplantation (especially the 3–6 months window period)

Reference [33]	PET/CT after HSCT (post-PET) was associated with PFS (*P* = 0.030). However, none of the assessed factors predicted OS.	This meant that PET may help guide subsequent clinical treatment decisions.

Reference [34]	PET results were associated with 3-year PFS [HR = 4.391, *P* = 0.001; HR = 7.607, *P* < 0.001] and OS (HR = 4.792, *P* = 0.008; HR = 26.138, *P* < 0.001).	PET results were a useful prognostic factor in patients undergoing HSCT.

**Table 3:** Statistics of 18F-FDG PET/CT diagnosis and prediction results after treatment.

References	Research results	Research conclusions
Reference [36]	Posttreatment assessment, significantly correlated with ΔSUV max (*p* = 0.04) but achieved a slightly significant correlation with deauville criteria (*p* = 0.055 and *p* = 0.058). Overall, 1, 3, and 5-year PFS were 95.7 ± 0.2, 89.6 ± 0.4, and 80.8 ± 0.7%, respectively.	Quantitative and visual assessment of IHP can be reliably used at the end of treatment

Reference [37]	FDG-PET/(CT) found 27.8% of additional lesions not detected by CT and/or MRI; 29.0% (95% CI: 14.0%–50.5) had a change in FDG-PET(/CT) result or guided treatment %) (I2 = 40.1%).	FDG-PET(/CT) was the most frequently studied imaging modality in patients with PTLD.

Reference [38]	The pooled sensitivity of F-18 FDG PET or PET/CT was 0.90, the overall specificity was 0.90, the positive likelihood ratio was 9.4, the negative likelihood ratio was 0.11, and the diagnostic odds ratio was 83.	F-18 FDG PET or PET/CT had high sensitivity and specificity for the detection of PTLD.

The article "PET/CT Evaluation of the Effect of Allogeneic Hematopoietic Stem Cell Transplantation in the Treatment of T-Cell Lymphoblastic Lymphoma" was published in 2022. Journal: Contrast Media Mol Imaging.

**Table 4:** Application limitations of ^18^F-FDG PET/CT.

Reference no.	Title	Research objective	Application limitations of ^18^F-FDG PET/CT
[36]	^18^F-FLT-PET/CT adds value to ^18^F-FDG-PET/CT for diagnosing relapse after definitive radiotherapy in patients with lung cancer. Results of a prospective clinical trial	It investigated the value of ^18^F-FLT-PET/CT and ^18^F-FDG-PET/CT in diagnosing recurrence of radiation cancer	The specificity of 18F-FLT-PET/CT and 18F-FDG-PET/CT in the diagnosis of cancer patients after recurrence was reduced, and the efficiency of single application was significantly lower than the effect of the combination of the two

[37]	Prognostic value of 2-deoxy-2-[^18^F]fluoro-D-glucose positron emission tomography/computed tomography after autologous hematopoietic stem cell transplantation in lymphoma using deauville scores	It aimed to evaluate 2-deoxy-2-[^18^F]fluoro-D-glucose ([^18^F]F-FDG) positron emission tomography (PET)/computed tomography (CT) in lymphoma autologous stem cell transplantation (ASCT)	Applicable time was limited.

[38]	Prognostic value of ^18^F-FDG PET/CT in T-Lymphoblastic lymphoma before and after hematopoietic stem cell transplantation	It was to evaluate the prognostic value of ^18^F-FDG PET/CT in patients with relapsed or refractory t-lymphoid transplantation (T-LBL) undergoing hematopoietic stem cell transplantation (HSCT).	Pre-PET failed to predict PFS and OS in T-LBL patients treated with HSCT.

[41]	Prediction of outcome in pediatric Hodgkin lymphoma based on interpretation of ^18^FDG-PET/CT according to DSUVmax, deauville 5-point scale and IHP criteria	It compared different interpretation methods of ^18^F-FDG PET/CT in predicting disease prognosis to determine the best method in this regard	Effective evaluation indicators for predicting disease prognosis were different before and after treatment, and further research was needed to find the best indicator

[42]	Performance of advanced imaging modalities at diagnosis and treatment response evaluation of patients with posttransplant lymphoproliferative disorder: a systematic review and meta-analysis	It aimed to evaluate the clinical performance of advanced imaging modalities in the diagnosis and treatment response assessment of PTLD patients after solid organ and hematopoietic stem cell transplantation	FDG-PET(/CT) was well-applied for detection, staging, and treatment evaluation, but has methodological flaws, false-negatives due to physiologic high background activity and early PTLD lesions, and false-positives due to inflammatory conditions

[43]	Diagnostic performances of F-18 FDG PET or PET/CT for detection of posttransplant lymphoproliferative disorder: a systematic review and meta-analysis	It aimed to investigate the diagnostic performance of F-18 FDG PET or PET or PET/CT for the detection of posttransplant lymphoproliferative disease (PTLD)	The scope of the study was limited and further large multicenter studies were needed to confirm

The article "PET/CT Evaluation of the Effect of Allogeneic Hematopoietic Stem Cell Transplantation in the Treatment of T-Cell Lymphoblastic Lymphoma" was published in 2022. Journal: Contrast Media Mol Imaging.

## Data Availability

The data used to support the findings of this study are available from the corresponding author upon request.
